The article "Systematic Pharmacology-Based Strategy to Explore the Mechanism of Bufei Huoxue Capsule in the Treatment of Chronic Obstructive Pulmonary Disease" was published in 2022. Journal: Evid Based Complement Alternat Med.

# Systematic Pharmacology-Based Strategy to Explore the Mechanism of Bufei Huoxue Capsule in the Treatment of Chronic Obstructive Pulmonary Disease

**DOI:** 10.1155/2022/1129567

**Published:** 2022-12-06

**Authors:** Liangtian Shi, Jun Yan, Yufeng Meng, Guishu Wang, Jianchao Du, Cuiling Feng

**Affiliations:** ^1^Beijing University of Chinese Medicine, Beijing 100029, China; ^2^Dongzhimen Hospital, Beijing University of Chinese Medicine, Beijing 100700, China; ^3^Peking University People' Hospital, Beijing 100044, China

## Abstract

**Objective:**

To explore the effects and mechanisms of Bufei Huoxue Capsule (BHC) on chronic obstructive pulmonary disease (COPD) based on network pharmacology.

**Methods:**

The effective components and related targets of BHC were collected by searching TCMSP, HERB, and ETCM databases, after which the related targets of COPD were obtained on GeneCards and OMIM databases. The common targets were imported into the STRING database and Cytoscape database to construct a target interaction network and screen core targets. Next, Gene Ontology (GO) and Kyoto Encyclopedia of Genes and Genomes (KEGG) pathway enrichment analyses were performed on the Metascape platform. According to the prediction results of network pharmacology, the action mechanism was further examined in an animal model of COPD. The pathological changes of lung tissue were observed by HE staining; goblet cells and mucus secretion in lung tissue were observed by AB-PAS staining, airway collagen deposition was observed by Masson staining, and the expression of NE, TGF-*β*1, P-EGFR/EGFR, P-ERK1/2/ERK1/2, P-JNK/JNK, and P-P38/P38MAPK protein was detected by Western blot analysis.

**Results:**

A total of 379 targets related to BHC and 7391 targets related to COPD were obtained, including 313 potential targets of BHC in treating chronic obstructive pulmonary disease, with JUN, AKT1, TNF, IL6, EGFR, MAPK1, and MAPK14 as the core targets. Through enrichment analysis, BHC may interfere with COPD by regulating the MAPK signal pathway, HIF-1 signal pathway, NF-*κ*B signal pathway, cAMP signal pathway, cGMP-PKG signal pathway, and so on. Animal experiments showed that the BHC could reduce airway inflammatory cell infiltration, inhibit airway epithelial goblet cell proliferation, reduce mucus secretion, and improve small airway collagen fiber deposition in COPD model rats. Besides, BHC could downregulate the protein expression of NE, TGF-*β*1, P-EGFR, P-ERK1/2, and P-P38MAPK.

**Conclusion:**

BHC can reduce airway inflammation, inhibit mucus hypersecretion, and improve airway remodeling by regulating the MAPK signal transduction pathway.

## 1. Introduction

Chronic obstructive pulmonary disease (COPD) is a common, preventable, and treatable disease characterized by persistent respiratory symptoms and airflow limitation, usually caused by airway and/or alveolar abnormalities due to exposure to noxious particles or gases [1]. As the third leading cause of death globally [2], COPD contributes to a substantial social and economic burden. Smoking is the primary risk factor for COPD [3, 4]. Passive smoking, known as environmental smoking, may also contribute to the development of COPD [4, 5]. The harmful particles in tobacco, lipopolysaccharide, and other stress may enter the lung to cause inflammation, which stimulates the increase of goblet cells, the increase in the volume of the submucous gland, and the high secretion of mucus in the lung. With repeated injury and repair, small airway stenosis, pulmonary parenchyma destruction, and lung structural changes occur, leading to persistent airflow limitation [6]. As a consequence, chronic inflammation [7], mucus hypersecretion [8], and airway remodeling [9] are the main pathological features of COPD.

The article "Systematic Pharmacology-Based Strategy to Explore the Mechanism of Bufei Huoxue Capsule in the Treatment of Chronic Obstructive Pulmonary Disease" was published in 2022. Journal: Evid Based Complement Alternat Med.

Pharmacological therapy for COPD mainly includes *β*2 agonists, anticholinergics, theophylline, glucocorticoids, antibiotics, expectorants, and antioxidant drugs [1]. The above drugs can improve clinical symptoms, reduce the risk of acute exacerbation, and improve patients' exercise endurance but cannot modify the long-term decline of lung function [1, 10]. In recent years, traditional Chinese medicine (TCM) treatment of COPD has been mostly based on deficiency, phlegm, and blood stasis, achieving promising results. Bufei Huoxue capsule, composed of *Radix Astragalus Hedysari* (milkvetch root), *Radix Paeoniae Rubra* (peony root), and *Fructus Psoraleae* (malaytea scurfpea fruit) according to the proportion of 2 : 2 : 1 is typically used to invigorate the lung, strengthen the spleen, consolidate the kidney, replenish qi, and activate blood circulation. By regulating the functions of the lung, spleen, and kidney, BFHX capsules can promote the operation of qi and blood, improve fluid metabolism, and improve the aspects of “deficiency, phlegm, and blood stasis.” Previous clinical studies have shown that BHC can relieve clinical symptoms in COPD patients, suppresses inflammatory injury of the lung, ameliorate pulmonary vascular hemodynamics, improve pulmonary function, and reduce the number of acute attacks [11, 12]. On the other hand, few patients treated with BHCs reported adverse events (AEs), such as elevated levels of ALT and AST; yet, after drug withdrawal and symptomatic treatment, the abnormal test indices returned to normal within two weeks. Also, no significant difference was observed in the incidence of adverse events between BFHX groups and other groups [13, 14]. Still, the exact mechanism through which BHC affects COPD is unclear.

The article "Systematic Pharmacology-Based Strategy to Explore the Mechanism of Bufei Huoxue Capsule in the Treatment of Chronic Obstructive Pulmonary Disease" was published in 2022. Journal: Evid Based Complement Alternat Med.

Network pharmacology analyses the action law of TCM compound prescription based on the theory of system biology constructs the drug-disease interaction network and reveals the action mechanism of TCM compound prescription on disease treatment [15]. In this study, we used network pharmacology to predict the core targets and pathways of BHC in the treatment of COPD and verify the regulation of the MAPK signal transduction pathway by animal experiments based on the previous rat model of COPD [16, 17] (Figure 1), so as to provide a scientific basis for the clinical application of BHC.

## 2. Materials and Methods

### 2.1. Network Pharmacology Research

#### 2.1.1. Collection of BFHX Potential Active Compounds and Corresponding Targets

Based on the TCM network pharmacology data analysis platform (TCMSP, https://old.tcmsp-e.com/tcmsp.php) [18], HERB database (http://drug.ac.cn) [19], and ETCM database (http://www.tcmip.cn/ETCM/) [20], the chemical constituents of BHC (*Radix Astragalus Hedysari*, *Radix Paeoniae Rubra,* and *Fructus Psoraleae*) were collected. All chemical components were substituted into the TCMSP database with oral bioavailability (OB) ≥ 30% and drug-likeness (DL) ≥ 0.18 as limiting conditions. The components which were not observed in the HERB database were required to meet the screening criteria of the Swiss ADME database (http://www.swissadme.ch) [21], in which gastrointestinal GI absorption was set as “high,” and DL items were set as “yes.” The components which were not observed in the ETCM database were required to meet the drug similarity level of “good” in this database. According to the above criteria, the potential active components of BHC were selected and substituted into the TCMSP database to find their corresponding targets. The chemical structure formula of chemical components without target information in the TCMSP database was downloaded; then, the PharmMapper database (http://lilab-ecust.cn/pharmmapper/index.html) [22] was used to predict the targets, with a normalized fit score ≥0.9 as the screening standard. Uniport database (https://www.uniprot.org) [23] was used to calibrate all targets, delete nonhuman target proteins, and obtain the final potential targets of BFHX. The herb-compound-target network was constructed and visualized using Cytoscape 3.8.2 software.

#### 2.1.2. Acquisition of COPD-Associated Targets

According to databases of OMIM (https://www.omim.org) [24] and GeneCards (https://www.genecards.org) [25], keywords such as “chronic obstructive pulmonary disease” and “COPD” were employed to search the COPD-related targets. The targets of the GeneCards database were selected based on Score ≥1, and all the targets of the OMIM database were collected. After removing the duplicate targets, COPD-related targets were eventually collected.

The article "Systematic Pharmacology-Based Strategy to Explore the Mechanism of Bufei Huoxue Capsule in the Treatment of Chronic Obstructive Pulmonary Disease" was published in 2022. Journal: Evid Based Complement Alternat Med.

#### 2.1.3. Screening the Related Targets of BFHX in the Treatment of COPD

The acquired targets of BFHX and COPD were imported to draw a Venn diagram using Venny 2.1 (https://bioinfogp.cnb.csic.es/tools/venny/) [26]. The intersections were obtained as the potential targets of BFHX in treating COPD.

#### 2.1.4. Construction of Protein-Protein Interaction (PPI) Network between BFHX and COPD

The above potential targets were imported into the STRING database (STRING, https://www. string-db.org) [27] to screen PPI network characteristic data, setting the species as “*Homo sapiens*” and threshold combined score > 0.95 as limiting conditions; discrete protein nodes were excluded. The obtained data were imported into Cytoscape software [28] for visual analysis. The major topological parameters were “degree value” and “combine-core value,” which were used to identify the key genes.

#### 2.1.5. Enrichment Analysis of GO Analysis and KEGG Pathway Based on the Intersection Targets

The potential target of BFHX in treating COPD was substituted into Metascape's online analysis platform (http://metascape.org) [29]. The enrichment analysis of Gene Ontology (GO) and Kyoto Encyclopedia of Genes and Genomes (KEGG) pathway was carried out. The relevant biological processes (BPs), cellular components (CCs), molecular functions (MFs), and signal pathways of the potential targets were imported into the WeChat analysis platform (http://www.bioinformatics.com.cn) [30] for visual analysis with [31] bubble diagrams.

### 2.2. Experimental Research

#### 2.2.1. Experimental Animals

A total of 40 SPF male Wistar rats weighing 200 ± 20 g were provided by Sibefu (Beijing) Biotechnology Co., Ltd., (license no.: SCXK (Beijing) 2018–0006). All the animals were housed in an environment with a temperature of 22 ± 1°C, a relative humidity of 50 ± 1%, a light/dark cycle of 12/12 hr, a given standard pellet, and clean drinking water. All animal studies were conducted in compliance with the regulations of the Peking University people's Hospital animal laboratory and conducted according to the Experimental Animal Ethics Committee of Peking University people's Hospital guidelines (approval no.: 2020PHE041).

#### 2.2.2. Experimental Drugs and Reagents

BHC (*Radix Astragalus Hedysari*, *Radix Paeoniae Rubra*, and *Fructus Psoraleae*) was provided by Guangdong Lei Yun Shang Pharmaceutical Co., Ltd. National Medicine Standard Z20030063. Theophylline sustained-release tablets were obtained from Guangzhou Maite Xinghua Pharmaceutical Co., Ltd. National Medicine Standard H44023791.

The article "Systematic Pharmacology-Based Strategy to Explore the Mechanism of Bufei Huoxue Capsule in the Treatment of Chronic Obstructive Pulmonary Disease" was published in 2022. Journal: Evid Based Complement Alternat Med.

The reagents for HE staining were provided by the Central Laboratory of Peking University people's Hospital. The other reagents were purchased as follows: AB-PAS staining kit (Beijing Solarbio Technology Co., Ltd., batch no. G1285), Masson staining kit (BestBio, batch no. BB-4422), rabbit polyclonal antibody NE (Abcam, batch no. ab21595), rabbit polyclonal antibody TGF-*β*1 (affinity, batch no. AF1027), rabbit polyclonal antibody EGFR (Proteintech, batch no. 18986-1-AP), rabbit monoclonal antibody phospho-EGFR (CST, batch no. 3777S), rabbit polyclonal antibody JNK (affinity, batch no. AF6319), rabbit polyclonal antibody phospho-JNK (affinity, batch no. AF3318), rabbit polyclonal antibody ERK1/2 (Proteintech, batch no. 11257-1-AP), rabbit monoclonal antibody phospho-ERK1/2 (CST, batch no. 4370S), rabbit monoclonal antibody P38-MAPK (CST, batch no. 8690S), rabbit polyclonal antibody phospho-P38-MAPK (affinity, batch no. AF4001).

#### 2.2.3. Animal Grouping, Modeling, and Intervention

After three days of adaptive feeding, rats were randomly divided into the following 4 groups: the normal control group (control), model group (COPD), Bufei Huoxue group (BFHX), and theophylline group (theophylline). The rat model of COPD was established by cigarette smoke exposure combined with airway instillation of LPS. The rats were smoked with a self-made smoke fumigation box. Each time, 8 cigarettes were lit to fume 10 rats, once a day for 30 min. The cigarette smoke exposure to the 28th day. The LPS powder was mixed with normal saline to get an LPS solution, with a concentration of 1 mg/mL. 200 *μ*L of LPS solution was dripped through the airway on the 1st, 11^th^, and 21st of the experiment, and the rats did not smoke on the drip day. The control group was not exposed to smoke and was not dripped with LPS solution. From the 21st day of modeling, the normal control group and model group were given 10 mL/kg of normal saline once a day for 40 days, the Bufei Huoxue group received a daily gavage of 0.42 g/kg BHC powder diluted into 10 ml/kg with distilled water for 40 days, and the theophylline group received a daily gavage of 0.02 g/kg theophylline sustained-release tablet powder diluted into 10 ml/kg with distilled water for 40 days.

#### 2.2.4. Pathological Observation by Hematoxylin-Eosin Staining (HE), Alcian Blue-Periodate Schiff Staining (AB-PAS), and Masson Staining (Masson)

On day 61 after modeling, all rats were anesthetized with 1% pentobarbital sodium at the dose of 50 mg/kg. After abdominal aortic blood was collected, the chest was open, the hilum of the right lung was tightened, and the left lung was collected, fixed in 4% paraformaldehyde solution, dehydrated, transparent, paraffin-impregnated, and embedded. Then, the paraffin tissue was cut into a 3 *μ*m section, dewaxed, and stained with the HE method. The morphology of lung tissues and airways was evaluated by Leica light microscope. AB-PAS was applied to detect goblet cells of the bronchial epithelium and mucus secretion; Masson staining was applied to detect collagen deposition in the airway. The images of lung tissues were captured by microscope.

The article "Systematic Pharmacology-Based Strategy to Explore the Mechanism of Bufei Huoxue Capsule in the Treatment of Chronic Obstructive Pulmonary Disease" was published in 2022. Journal: Evid Based Complement Alternat Med.

#### 2.2.5. Expression of NE, TGF-*β*1, P-EGFR/EGFR, P-ERK1/2/ERK1/2, P-P38/P38 MAPK, and P-JNK/JNK Protein in Lung Tissue Detected by Western Blot Analysis

A lung tissue (30 mg) of the rats was extracted by RIPA buffer containing protease inhibitors and centrifuged to extract total proteins. The protein content was determined by the Bradford assay (BCA) method, mixed with 4 × SDS loading buffer, and denatured at 96°C for 5 min. The same amount of extracted fresh proteins was separated by SDS-PAGE electrophoresis and transferred to the PVDF membrane. The membrane was blocked with 5% skimmed milk powder for 60 min. The PVDF membranes were incubated with primary antibodies (NE 1 : 1000, TGF-*β*1 1 : 500, EGFR 1 : 2000, P-EGFR 1 : 1000, P-ERK1/2 1 : 1000, ERK1/2 1 : 1000, P-P38-MAPK 1 : 2000, P38-MAPK 1 : 1000, P-JNK 1 : 1000, and JNK 1 : 1000) at 4°C overnight. Afterward, the PVDF membranes were incubated with HRP-conjugated secondary antibody at room temperature for 60 min. At last, the PVDF membranes were developed with an ECL reagent and photographed by the gel-imaging system. Image J image analysis software was used to measure the image's average optical density. The expression of the target protein was determined by the optical density value of the target band/the optical density value of the internal reference band.

#### 2.2.6. Statistical Analysis

SPSS22.0 was adopted for statistical analysis. The measurement data were expressed by mean ± standard deviation. The statistical differences between groups were determined by one-way analysis of variance (ANOVA). *P* < 0.05 indicated that the difference was statistically significant.

## 3. Results

### 3.1. Target Prediction of BFHX in the Treatment of COPD by Network Pharmacology Research

#### 3.1.1. BFHX Potential Active Compounds and Corresponding Targets

A total of 97 kinds of effective chemical constituents were screened from 3 herbs of BFHX (*Radix Astragalus Hedysari*, *Radix Paeoniae Rubra*, and *Fructus psoraleae*), including 35 kinds of *Radix Astragalus Hedysari*, 42 kinds of *Radix Paeoniae Rubra*, and 20 kinds of *Fructus psoraleae*. Six kinds of repeated chemical constituents were screened, and 91 effective chemical constituents were identified. The related targets were collected, and the repeated targets were eliminated. Finally, 379 targets were obtained. The herb-compound-target (H-C-T) was constructed by Cytoscape (Figure 2). The network consists of 91 compound nodes, 379 gene nodes, and 2105 edges, which indicates that not only the composition of BFHX is complex and multitarget, but there is also a close relationship between composition and target.

The article "Systematic Pharmacology-Based Strategy to Explore the Mechanism of Bufei Huoxue Capsule in the Treatment of Chronic Obstructive Pulmonary Disease" was published in 2022. Journal: Evid Based Complement Alternat Med.

#### 3.1.2. Potential Targets of BFHX in the Treatment of COPD

A total of 7391 targets related to COPD were obtained by searching the OMIM database and GeneCards. Venn diagram was drawn using Venny 2.1 (Figure 3). There are 313 potential targets of BFHX in the treatment of COPD.

#### 3.1.3. Screening of Core Targets of BFHX in the Treatment of COPD and Construction of PPI Network

The potential targets of BFHX in the treatment of COPD were imported into the STRING database to construct the PPI network (Figure 4). According to the order of degree values, the higher the degree value, the larger the node, and the closer to the center. Consequently, the top 15 targets were: JUN, AKT1, HSP90AA1, SRC, TP53, TNF, IL6, RELA, ESR1, EGFR, MAPK1, GRB2, MAPK14, MYC, and FOS. These targets were the core targets of BFHX in the treatment of COPD.

#### 3.1.4. Enrichment Analysis of the Potential Targets of BFHX in the Treatment of COPD

Metascape database was adopted to analyze the GO function and KEGG pathway enrichment of the potential targets of BFHX in treating COPD (Figure 5). The top 20 cellular signaling pathways are as follows: cancer pathways in cancer, lipid, and atherosclerosis, signaling pathway in diabetic complications, chemical carcinogenesis-receptor activation, chemical carcinogenesis-reactive oxygen species, MAPK signaling pathway, HIF-1 signaling pathway, insulin resistance, NF-*κ*B signaling pathway, platinum drug resistance, pathways of neurodegeneration-multiple diseases, thyroid hormone signaling pathway, transcriptional misregulation in cancer, acute myeloid leukemia, malaria, calcium signaling pathway, rheumatoid arthritis, progesterone-mediated oocyte maturation, cAMP signaling pathway, and cGMP-PKG signaling pathway.

The top 20 biological processes in GO enrichment analysis include response to the hormone, response to xenobiotic stimulus, cellular response to lipid, response to an inorganic substance, response to wounding, positive regulation of cell motility, response to cytokine, positive regulation of cell death, response to decreased oxygen levels, reproductive structure development, response to extracellular stimulus, positive regulation of protein phosphorylation, response to a steroid hormone, gland development, response to growth factor, regulation of cell adhesion, blood circulation, aging, response to alcohol, and protein phosphorylation.

The article "Systematic Pharmacology-Based Strategy to Explore the Mechanism of Bufei Huoxue Capsule in the Treatment of Chronic Obstructive Pulmonary Disease" was published in 2022. Journal: Evid Based Complement Alternat Med.

The top 20 cell components in GO enrichment analysis include membrane raft, vesicle lumen, receptor complex, side of the membrane, transcription regulator complex, extracellular matrix, focal adhesion, postsynapse, perinuclear region of cytoplasm, dendrite, protein kinase complex, endoplasmic reticulum lumen, lytic vacuole, apical part of cell, outer organelle membrane, blood microparticle, cytoplasmic side of membrane, endocytic vesicle, serine-type peptidase complex, and peptidase inhibitor complex.

The top 20 molecular functions in GO enrichment analysis include nuclear receptor activity, kinase binding, protein kinase activity, oxidoreductase activity, protein domain-specific binding, lipid binding, protein homodimerization activity, cytokine receptor binding, carboxylic acid binding, antioxidant activity, serine hydrolase activity, heme binding, G protein-coupled amine receptor activity, amide binding, phosphatase binding, scaffold protein binding, phosphoprotein binding, protease binding, integrin binding, and NADP binding.

#### 3.1.5. The Role of the MAPK Signaling Pathway in the Treatment of COPD by BFHX

Through network pharmacology research, MAPK1 and MAPK14 were obtained as important targets of BFHX for treating COPD. Using KEGG pathway enrichment analysis, the MAPK signaling pathway was judged as the core signaling pathway of BFHX for treating COPD. The MAPK signaling pathway is shown in Figure 6. MAPK signaling pathway includes classical MAP kinase pathway, JNK, and p38 MAP kinase and ERK5 pathways. The growth factors (GFs) combined with receptor tyrosine kinase (RTK) can activate RAS and recruit Raf (MAP3K) on the cell membrane. Activated Raf then phosphorylates and activates MEK (MAP2k). The threonine and tyrosine residues of MEK phosphorylate and activate ERK, which enters the nucleus and causes the transcription of downstream signals, regulating the proliferation and differentiation of cells. In addition, inflammatory factors, TGF*β*, lipopolysaccharide, and other stress can activate JNK and P38 MAP kinase pathways. The above stresses activate MAP3K (including MEKK1, MEKK2, MEKK3, and ASK), and then the phosphorylated MAP3K activates MAP2K (MEKK4, MEKK6, MEKK7, etc.). The threonine proline tyrosine motifs of MAP2K phosphorylate and activate JNK and P38. Activated JNK and P38 can interact with downstream nuclear and cytoplasmic proteins, leading to the proliferation, differentiation, inflammation, and apoptosis of cells. Current studies have shown that ERK1/2, P38 MAPK, and JNK are able to be activated in COPD, release inflammatory factors, promote mucin expression, and regulate cytokine transcription [1].

The article "Systematic Pharmacology-Based Strategy to Explore the Mechanism of Bufei Huoxue Capsule in the Treatment of Chronic Obstructive Pulmonary Disease" was published in 2022. Journal: Evid Based Complement Alternat Med.

### 3.2. Experimental Study on the Effect of BFHX on COPD Based on MAPK Signal Pathway

#### 3.2.1. HE Staining to Observe the Pathological Changes in Rat Lung Tissue

The lung tissues of each group were stained with HE. As shown in Figure 7, in the normal control group, the airway epithelium was intact with a small amount of cilia adhesion, no shedding, uniform airway smooth muscle, no hyperplasia, no hyperemia, no inflammatory cell infiltration, no glandular hyperplasia, and complete alveolar structure. Compared with the normal control group, the model group had thickened airway epithelium, adhered and shredded cilia, thickened airway smooth muscle, inflammatory cell infiltration, destructed alveolar structure, and widened alveolar septum. In the BFHX and theophylline groups, the airway epithelium was regularly arranged, the lodging and shedding of cilia were improved, the alveoli were relatively intact, the alveolar fusion was reduced, and the infiltration of inflammatory cells and red blood cells was reduced.

#### 3.2.2. AB-PAS Staining Showing Airway Epithelial Goblet Cells and Mucus Secretion

AB-PAS staining was performed on paraffin sections of rat lung tissues (Figure 8). In the normal control group, there was no goblet cell metaplasia in the airway epithelium, columnar epithelial cells were regularly arranged, and a small amount of blue-stained mucins could be observed in the submucosa. Compared with the normal control group, many blue-stained goblet cells could be observed in the airway epithelium of the model group, and the blue-stained mucins in the submucosa were more obvious. In the BFHX group and theophylline group, goblet cells and blue-stained mucin were significantly reduced.

#### 3.2.3. Masson Staining to Observe the Collagen Deposition in the Airway

The paraffin sections of rat lung tissues were stained with Masson. In the normal control group, a small amount of blue-stained collagen fibers and thin and uniform muscle fibers could be observed between the airway epithelium and submucosa. Compared with the normal control group, many blue-stained collagen fibers could be observed in the airway epithelium and submucosa of the model group, and part of the red smooth muscle was destroyed by inflammatory cells. In the BFHX and theophylline groups, the blue collagen fibers between airway epithelium and submucosa decreased significantly, and the red smooth muscle was thin and uniform without rupture (Figure 9).

The article "Systematic Pharmacology-Based Strategy to Explore the Mechanism of Bufei Huoxue Capsule in the Treatment of Chronic Obstructive Pulmonary Disease" was published in 2022. Journal: Evid Based Complement Alternat Med.

#### 3.2.4. Expression of NE, TGF-*β*1, P-EGFR/EGFR, P-ERK1/2/ERK1/2, P-P38/P38 MAPK, and P-JNK/JNK Protein in Lung Tissue by Western Blot Analysis

To detect the effect of BFHX on proteins related to MAPK signal transduction pathway-related molecules, we measured the proteins of NE, TGF-*β*1, EGFR, P-EGFR, ERK1/2, P-ERK1/2, JNK, P-JNK, P38, and P-P38 in lung tissues of rats in each group detected by Western blot analysis. The Image J image analysis software was used to calculate the optical density of bands. NE/GAPDH, TGF-*β*1/GAPDH, P-EGFR/EGFR, P-ERK/ERK, P-JNK/JNK, and P-P38/P38 were adopted as quantitative indexes for quantitative analysis. Compared with the normal control group, the expressions of NE, TGF-*β*1, P-EGFR/EGFR, P-ERK/ERK, and P-P38/P38 in the model group were significantly increased (*P* < 0.05), but there was no significant difference in the expression of P-JNK/JNK (*P* > 0.05). Compared with the model group, the expressions of NE, TGF-*β*1, P-EGFR/EGFR, P-ERK/ERK, and P-P38/P38 in the BFHX group and theophylline group decreased (*P* < 0.05), and the expression of P-JNK/JNK in the theophylline group decreased compared with the model group (*P* < 0.05). There was no significant difference in protein expression between the BFHX group and the theophylline group (*P* > 0.05) (Figure 10).

## 4. Discussion

COPD is a chronic inflammatory disease of the airway, pulmonary parenchyma, and pulmonary vessels caused by multiple factors [32]. The pathogenesis of COPD is complex and still not fully understood. In this study, we screened the key components, targets, and pathways of BFHX in treating COPD, constructed the PPI network, and obtained the targets' KEGG and GO enrichment analysis by network pharmacology. The results showed that JUN, AKT1, EGFR, MAPK1, MAPK14, and more were regarded as the core targets of treating COPD by BFHX. The effects of BFHX in COPD were complex, involving multitargets and multiple pathways; the main biological processes included a response to xenobiotic stimulus, response to cytokine, response to growth factor, regulation of cell adhesion and protein phosphorylation, through key pathways such as cancer pathways in cancer, lipid, and atherosclerosis, signaling pathway in diabetic complications, chemical carcinogenesis-receptor activation, MAPK signaling pathway, among which MAPK signaling pathway showed an important role. Therefore, the MAPK signaling pathway may provide an idea and direction for experimental animal research in treating COPD with BFHX.

Cigarette smoke is the most common cause of COPD [1]. LPS, as a stressor, can activate macrophages and epithelial cells, promote the release of cytokines and inflammatory mediators, and cause a series of organism reactions [33]. Chronic inhalation of irritants, including cigarette smoke and LPS, enter the lungs through the respiratory tract and activate an innate immune response, which results in the activation of airway epithelial cells, macrophages, and neutrophils, as well as the activation of pulmonary inflammation. Airway epithelial cells and macrophages release multiple chemotactic factors, which attract neutrophils, monocytes, and T lymphocytes and lead to adaptive immunity. Activated inflammatory and structural cells release multiple inflammatory mediators [34, 35]. Various inflammatory cells, cytokines, and mediators interact together to participate in the inflammatory process, leading to protease release, stimulating mucus hypersecretion, and breaking down the connective tissue in the lung parenchyma. In addition, several inflammatory cells, such as epithelial cells and macrophages, release fibrogenic mediators that activate fibroblasts leading to small airway fibrosis. In our previous studies, we established the rat model of COPD by cigarette smoke exposure combined with airway instillation of LPS [16, 17]. The results showed that the rat model of COPD established by this method conformed to the pathological changes of human COPD. In this study, we successfully replicated the previous rat model of COPD. The results of pathological staining demonstrated airway epithelial thickening, adhering and shredded cilia, thickening of airway smooth muscle, a proliferation of glandular, infiltration of inflammatory cells, alveolar structure destruction, alveolar collapse, alveolar fusion, alveolar septum thickening, pulmonary interstitial inflammatory cells, and red blood cell infiltration. The pathological manifestations were consistent with the pathological features of airway inflammation, mucus hypersecretion, and airway remodeling in COPD. Importantly, BFHX or theophylline improved histopathological injury, reduced inflammatory cell infiltration, inhibited mucus hypersecretion, and ameliorated collagen deposition.

The article "Systematic Pharmacology-Based Strategy to Explore the Mechanism of Bufei Huoxue Capsule in the Treatment of Chronic Obstructive Pulmonary Disease" was published in 2022. Journal: Evid Based Complement Alternat Med.

NE, TGF-*β*1, and EGF are released by neutrophils, macrophages, epithelial cells, and fibroblasts, and have an important role in airway inflammation, mucus hypersecretion, and airway remodeling in COPD. NE, an important enzyme associated with the inflammation of COPD, belongs to the chymotrypsin superfamily of serine proteases [36]. Studies have observed elevated NE in the serum and sputum of COPD patients [37, 38]. In addition to degrading elastase and dissolving other proteins, NE stimulates mucin production and secretion by the EGFR cascade [39], which can aggravate the inflammatory response and contribute to airway obstruction in COPD patients [40]. Furthermore, NE can stimulate airway smooth muscle proliferation and regulate airway remodeling by promoting the expression of TGF-*β*1. In the present study, a significant increase in the ratio of NE was detected in COPD lung tissues, while NE was reduced in the BFHX and theophylline groups. The results indicated that BFHX and theophylline could effectively reduce the activation of NE, which contributes to the mitigation of airway inflammation, mucus hypersecretion, and airway remodeling.

EGFR is one of the key molecules implicated in the expression of chemokines and mucins, and goblet cell metaplasia. In the surface epithelium of lung tissue, EGFR can be activated by cigarette smoke and several structurally related ligands like epidermal growth factor (EGF) [41], transforming growth factor-*α* (TGF-*α*) [42], amphiregulin (AR) [43], betacellulin (BTC) [44], and epiregulin [45]. Activated EGFR is phosphorylated and triggers signal transduction cascades, such as MAPK, Akt, and JNK pathways, which regulate cell migration, adhesion, differentiation, and proliferation [46], and promote excess mucin synthesis [47, 48]. Takeyama et al. observed that exposure to cigarette smoke leads to mucus hypersecretion and increased goblet cells through activation of the EGFR tyrosine phosphorylation [49, 50]. In this study, we observed increased p-EGFR in COPD rats compared with the control group, whereas it decreased after administration of BFHX and theophylline.

TGF-*β*1 is the most abundant isoform of the transforming growth factor superfamily [51], sourced from structural cells and inflammatory cells in the airway [52, 53], affecting cell proliferation, differentiation, and inflammation. It can mediate the proliferation and transformation of fibroblasts and airway smooth muscle cells [54, 55]. It can also promote the formation of elastin [56–58], help repair damage to the lungs, and exert an essential role in airway remodeling [59, 60]. As downstream signal proteins of TGF-*β*1, Smad proteins, phosphatidylinositol 3-kinase (PI3K), calmodulin-dependent protein kinase II, c-Ab l, and the MAPKs (ERK, JNK, and p38) regulate many cellular functions, including cell activation and proliferation [61]. Studies in patients with COPD have shown that TGF-*β*1 expression is upregulated in the airway epithelium and that TGF-*β*1 induces epithelial-mesenchymal transition (EMT) in the bronchial epithelial cells [62–64]. Moreover, Godinas et al. claimed that the levels of TGF-*β*1 are proportional to the severity of airway obstruction [65]. In our study, the level of TGF-*β*1 in COPD rats was significantly increased compared with the control group. After treatment with BFHX or theophylline, the results displayed a decrease in the expression of TGF-*β*1.

The article "Systematic Pharmacology-Based Strategy to Explore the Mechanism of Bufei Huoxue Capsule in the Treatment of Chronic Obstructive Pulmonary Disease" was published in 2022. Journal: Evid Based Complement Alternat Med.

MAPKs (mitogen-activated protein kinases) are serine-threonine protein kinases in cells, among which ERK1/2, JNK, and p38MAPK are the most studied subgroups. MAPK signaling cascade reaction can be activated by cigarette smoke, LPS, and cytokines (such as NE, TGF-*β*1, and EGFR) and promote cell proliferation, differentiation, apoptosis, and inflammation [66], which induces airway inflammation [67, 68], mucus hypersecretion [69], and airway remodeling [70, 71] (Figure 11). Grace et al. reported that the activated MAPKs translocate into the nucleus, where they activate transcription factors, leading to the transcription of genes for inflammatory cytokines [69]. Shin In-Sik reported that the expression of MUC5AC leading to mucus hypersecretion is mediated by EGFR, where the phosphorylation of MAPKs is a critical step [72]. Wang et al. observed that the reduction of airway remodeling in the COPD rat model induced by cigarette smoke and LPS is attributed to the inhibition of TGF-*β*1, which may be affected by negatively regulating phosphorylation of p38 MAPK [73]. Therefore, suppressing MAPK phosphorylation may be a therapeutic approach that inhibits inflammation, mucus hypersecretion, and airway remodeling in COPD. In this study, the MAPK pathway induced by NE, EGFE, and TGF-*β*1 activated the phosphorylation of ERK1/2, P38 MAPK, and JNK raised in COPD rats. Also, treatment with BFHX or theophylline effectively blocked the rise in phosphorylation of ERK1/2 and P38 MAPK. However, JNK phosphorylation does not seem to be activated in the two groups. These findings indicate that BFHX significantly reduces the expression of NE, EGFR, and TGF-*β*1 by suppressing the phosphorylation of MAPK, particularly ERK1/2 and P38 MAPK.

According to TCM theory, COPD is mainly caused by lung-spleen-kidney qi deficiency and phlegm-blood stasis obstruction. The therapy of “tonifying lung-spleen-kidney, supplementing qi, activating blood, and resolving phlegm” is wildly used for treating COPD [74]. BHC is composed of *Radix Astragalus Hedysari*, *Radix Paeoniae Rubra*, and *Fructus psoraleae*, with effects of “tonifying lung-spleen-kidney, supplementing qi and activating blood” [75]. Although these herbs cannot efficiently “resolve phlegm,” they can improve fluid metabolism and participate in resolving phlegm by regulating the functions of the lung, spleen, and kidneys. Recently, BHC was widely adopted in the clinic and showed beneficial effects on COPD patients [76] by improving clinical symptoms such as cough, expectoration, and dyspnea, reducing the number of acute attacks, downregulating the level of inflammatory factors, and improving lung function. Previous experimental studies [13, 14] showed that BHC had an effect on improving lung function, reducing pulmonary inflammation, inhibiting mucus hypersecretion, and ameliorating airway remodeling in COPD rats; however, the relevant mechanism remains unclear. This study copied the previous rat model of COPD by cigarette smoke exposure combined with intratracheal instillation of LPS. Morphology results demonstrated that BHC could improve histopathological injury, reduce inflammatory cells infiltration, inhibit mucus hypersecretion, and ameliorate collagen deposition. In addition, the network pharmacology showed that the MAPK pathway is a core signaling pathway for the treatment of COPD with BFHX. In further investigation of mechanisms, we observed that BHC had an effect on inhibiting phosphorylation of the MAPK signaling pathway, an approach that inhibits inflammatory, mucin expression, and fibroblast proliferation in COPD.

The article "Systematic Pharmacology-Based Strategy to Explore the Mechanism of Bufei Huoxue Capsule in the Treatment of Chronic Obstructive Pulmonary Disease" was published in 2022. Journal: Evid Based Complement Alternat Med.

In addition, the results of network pharmacology research suggested a complex network system composed of many components, multiple targets, and diverse pathways in the treatment of COPD by BFHX. The active components in BHC may play pivotal roles in anti-COPD through the core targets such as JUN, AKT1, HSP90AA1, SRC, TP53, TNF, IL6, RELA, ESR1, EGFR, MAPK1, GRB2, MAPK14, MYC, and FOS. Among them, JUN and AKT interact most closely with other proteins, which indicates that their binding function is strongly associated with COPD. However, according to the results of KEGG pathway enrichment, the MAPK signaling pathway is closely related to COPD and has been widely studied. Therefore, this study focuses more on the MAPK signaling pathway in treating COPD with BHC. However, as core targets, JUN and AKT may be chemical cores to continue with further studies.

## 5. Conclusion

This study demonstrated that BFHX could effectively reduce pulmonary inflammation, inhibit airway mucus hypersecretion, and improve airway remodeling in COPD rats. The mechanism may be achieved by regulating of MAPK signaling pathway. In addition, the results of network pharmacology research suggested a complex network system composed of many components, multiple targets, and diverse pathways in the treatment of COPD by BFHX. Therefore, BFHX can be a therapeutic method for COPD. Still, other possible mechanisms must be considered and further explored.

## Figures and Tables

**Figure 1:** Study flowchart.

**Figure 2:** H-T-C network. The herbs are marked as green, the compounds are marked as red, the repeated compounds are marked as purple, and the targets are marked as blue, HQ: *Radix Astragalus Hedysari*, CS: *Radix Paeoniae Rubra*, and BGZ: *Fructus psoraleae*.

The article "Systematic Pharmacology-Based Strategy to Explore the Mechanism of Bufei Huoxue Capsule in the Treatment of Chronic Obstructive Pulmonary Disease" was published in 2022. Journal: Evid Based Complement Alternat Med.

**Figure 3:** Potential targets of BFHX in treating COPD by Venn diagram.

**Figure 4:** PPI network of targets for BFXU in the treatment of COPD.

**Figure 5:** KEGG and GO enrichment analysis of the targets for BFHX in treating COPD.

**Figure 6:** MAPK signaling pathway (modified from hsa04010. BFHX-COPD target is marked pink).

**Figure 7:** HE staining of airways and alveoli: (a) control group, (b) COPD group, (c) BFHX group, and (d) theophylline group. The nucleus is colored blue-purple, while the red blood cells, cytoplasm, and extracellular matrix are red ×400.

**Figure 8:** AB-PAS staining of airways: (a) control group, (b) COPD group, (c) BFHX group, and (d) theophylline group. Airway epithelial goblet cells are colored in blue, and pseudostratified ciliated columnar epithelial cells in purple ×400.

**Figure 9:** Masson staining of airways: (a) control group, (b) COPD group, (c) BFHX group, and (d) theophylline group. Collagen fibers are blue, while muscle fibers, cytoplasm, and red blood cells are red ×400.

**Figure 10:** Expression of NE, TGF-*β*1, P-EGFR/EGFR, P-ERK1/2/ERK1/2, P-P38/P38 MAPK, and P-JNK/JNK protein in lung tissue. Compared with the control group,  ^*∗*^*P* < 0.05; compared with the model group,  ^#^*P* < 0.05.

**Figure 11:** Mechanism of the MAPK signaling pathway in treating COPD with BFHX.

## Data Availability

The images of this study are included within the article. The data used to support the findings of this study are available from the corresponding author upon request.
